The article "Children’s physical activity level and sedentary behaviour in Norwegian early childhood education and care: effects of a staff-led cluster-randomised controlled trial" was retracted in 2024. Reasons: results that could not be reproduced; errors in the methods; unreliable results or conclusions; concerns about the data.

# Children’s physical activity level and sedentary behaviour in Norwegian early childhood education and care: effects of a staff-led cluster-randomised controlled trial

**DOI:** 10.1186/s12889-020-09725-y

**Published:** 2020-11-04

**Authors:** Eivind Andersen, Steinar Øvreås, Kari Anne Jørgensen, Janne Borch-Jenssen, Thomas Moser

**Affiliations:** 1 Faculty of Humanities, Sports and Educational Science, University of South-Eastern Norway, Horten, Norway; 2 Sandefjord Municipality, Sandefjord, Norway

**Keywords:** ECEC, RCT, Children, Physical activity, Sedentary time

## Abstract

**Background:**

A growing body of evidence suggest that the children’s physical activity (PA) level in early childhood education and care (ECEC) settings are insufficient. Since most children attend ECEC settings for many hours on most days of the week, and these institutions reach children across the socioeconomic spectrum, the ECEC settings may serve as an ideal avenue for increasing physical activity level, reduce sedentary time and enhance the overall health of young children. This paper investigates the effectiveness of the “Active Kindergarten – Active Children” study to increase children’s PA level and reduce sedentary time within the ECEC setting.

**Methods:**

Accelerometers were used to asses PA and sedentary time. A total of 116 three to four-year olds took part in a randomised controlled trial in 11 ECEC settings. Participants were cluster-randomised, by ECEC setting, to either a 12 week staff-led and expert-supported intervention or a waiting list control group.

**Results:**

The intervention group increased time spent in moderate- and vigorous intensity PA by 10 min/day (95% CI = 3, 18; *P* = 0.01), took 1909 more steps per day (95% CI = 1130, 2688; *P* < 0.01) and reduced sedentary time with 14 min/day (95% CI = − 27, − 1; *P* = 0.04) compared to the control group. The intervention group had a 2.4 higher odds (95% CI = 1.05, 5.7; *P* = 0.04) of meeting the PA recommendations compared to the control group at follow-up.

**Conclusions:**

Our results show that a flexible staff-led and expert-supported multicomponent PA intervention can increase total PA level, moderate- and vigorous intensity PA and reduce time spent sedentary in three to four-year old children during their stay in ECEC settings.

**Trial registration:**

The trial was retrospectively registered on September 19, 2020 and available online at ClinicalTrials.gov: No. NCT04555746.

## Background

A growing body of evidence suggest that the children’s physical activity (PA) level in childhood education and care (ECEC) settings are insufficient [1, 2]. Moreover, sedentary behaviour, defined as any waking behaviour characterized by an energy expenditure ≤1.5 metabolic equivalents, while in a sitting, reclining, or lying posture [3], is highly prevalent [4] and has been identified as detrimental to children’s health [5]. Although many children have healthy and active lifestyles, there seems to be a relatively large group of children with a low PA level [6]. In turn, this could lead to negative developmental effects such as low fitness level, weak motor skills and obesity [7]. This is especially worrying because it is known that PA level often tracks from childhood into adulthood [8, 9]. Thus, early intervention is crucial, given that PA plays a pivotal role in children’s overall health and is associated with many positive health outcomes, including physical fitness [10], cardiovascular health [11], bone health [12] and psychosocial and cognitive development [12, 13].

The article "Children’s physical activity level and sedentary behaviour in Norwegian early childhood education and care: effects of a staff-led cluster-randomised controlled trial" was retracted in 2024. Reasons: results that could not be reproduced; errors in the methods; unreliable results or conclusions; concerns about the data.

PA levels has been found to be highly variable among children in ECEC settings [14, 15], and may therefore have great potential for effective interventions. Furthermore, since most children attend ECEC settings for many hours on most days of the week [16], and these institutions reach children across the socioeconomic spectrum, the ECEC settings may serve as an ideal avenue for increasing PA level, reduce sedentary time and enhancing the overall health of young children. Yet, early childhood educators identify parents rather than themselves as persons responsible for promoting children’s PA [17], and may assume that young children receive adequate PA throughout the week, regardless of activities during their stay in the ECEC setting [18]. Thus, intervening with children and staff in ECEC settings, to equip them with the knowledge, abilities and motivation to promote PA in children during their time in the ECEC, may provide substantial public health benefits [19].

In earlier studies, PA interventions conducted in ECEC settings [20, 21], have only shown small to moderate effects and were rather inconsistent across studies [20–23]. Most PA interventions that have been implemented in ECEC settings are structured programs developed by PA experts and delivered by staff alone or with great influence of trained research personnel [24]. In some studies, staff-led interventions have shown to be less effective in increasing PA compared to interventions implemented by PA experts [24, 25]. Similar findings have emerged regarding intervention effects on fundamental movement skills [26]. The main explanation for lower efficiency of staff led interventions may be that PA experts have more knowledge and competencies regarding this issue [26, 27]. In order to succeed with staff-led programs the need for multiple staff training sessions and maximizing the number of trained staff has been emphasized [25, 28].

The article "Children’s physical activity level and sedentary behaviour in Norwegian early childhood education and care: effects of a staff-led cluster-randomised controlled trial" was retracted in 2024. Reasons: results that could not be reproduced; errors in the methods; unreliable results or conclusions; concerns about the data.

Recently, several reviews have summarized the body of knowledge regarding various aspects of the contexts and prerequisites for PA in different kinds of out of home services for children in preschool age [28–30]. In a review including 34 studies, Hnatiuk at al. (2019) [30] revealed small, but positive and significant intervention effects only for children’s (≤ 5 years) moderate- to vigorous intensity PA (MVPA) but not light intensity PA. Based on their findings, the authors recommend interventions tailored to the target group, where cultural considerations, community needs and the provision of ongoing support should have a key role. Furthermore, they also conclude that daily structured PA sessions, integrated as part of the everyday activities in the institutions (routines) and delivered through a hands-on approach, will most likely contributed to increase children’s MVPA. Finally, Hnatiuk and colleagues claim that one should strive to influence the practices of both parents and staff as well as assessing and documenting changes in their PA levels, in order to illuminate the importance of their behaviour on children’s activity levels.

Jones et al. 2019 [28] conducted a review of 24 PA interventions in childcare mostly targeting children between three and 5 years of age where staff was participating in professional development either before or during the intervention period and providing children with opportunities for additional PA. Less than half of the included studies, caused positive effects on children’s PA level. For further intervention studies in ECEC the authors provided four recommendations, two of which were based on the papers included in the review and two based on evidence “from broader ECEC literature” (p. 8). Firstly, there is a need for high-quality professional development prior to and during the intervention, and, secondly, the necessity of “Interventions that are ‘outside the box’” (p. 8) in terms of e.g. blended professional development, the role of technology, targeting health, well-being and activity levels of the educators, focus on PA learning experiences, outdoor marking, and energy breaks and integration of interventions in the institutions daily routines. The third and broader based recommendation addresses the importance of developing meaningful and trustworthy cooperation and relationships between staff and researchers [31]. The fourth and final recommendation focuses on the ECEC environment as a key factor for providing good opportunities for PA and, thus, should be increasingly emphasized regarding future interventions.

The article "Children’s physical activity level and sedentary behaviour in Norwegian early childhood education and care: effects of a staff-led cluster-randomised controlled trial" was retracted in 2024. Reasons: results that could not be reproduced; errors in the methods; unreliable results or conclusions; concerns about the data.

A missing perspective in recent studies focusing on PA interventions in ECEC settings might be that they may not fully take into account the fact that ECEC teaching professions practice has become increasingly complex due to growing multi-diverse societies and multiple components related to working conditions [32]. Thus, top-down approaches and standardized solutions (programs) will possibly be harder to implement in an ever more diverse environment in terms of individual, social, cultural and physical differences within and between institutions. Therefore, it might be a suitable approach to establish an organizational and collaborative learning processes, a community of professional learning, to improve and maintain the staffs’ competence [28, 32, 33]. This means to contextualize pedagogical practice through continuous negotiation and reflection between staff members and through collective responsibility for improvement of practice, instead of purely implementing structured programs developed by external experts. While expert delivered interventions seem to be best suited for effect studies, “real-world” approaches implemented by preschool teachers may have a greater potential for developing a sustainable and improved long-term practice.

The current study therefore suggests a dialogical and bottom up approach that will take into account differences within and between local ECEC settings such as child group characteristics, staffs’ competencies and personal preferences and practices for sustainable implementation, differencies in the physical indoor and outdoor environments, as well as available equipment to promote physically active play [34]. Interventions that can be adapted to specific circumstances within an organization while maintaining overall fidelity are more likely to be successful [34]. Hence, the theoretical frame of the current intervention is based on Wenger’s theory on Communities of Practice (COP) [35]. Crucial for this theoretical perspective is the idea that organizations are learning communities sharing competence and experiences to develop new practices. Trusting in the staff’s professionalism and their knowledge about and sensitivity towards the individual child and the child groups as well as their awareness regarding barriers and possibilities in terms of environment and equipment. COP includes three modes of belongings; engagement, imagination and alignment. Engagement is active participating in the practice revealing needs for learning and changes, and establishing collective development of the organization. Imagination connects to the staff’s visions and their experience of meaning regarding the intervention, as well as their understanding of the purpose. Alignment is about the commitment to the entire project. To achieve positive changes based on COP these types of belonging has to be linked to particular processes such as the establishment of mutual engagement over time to promote changes, self-awareness and reflection concerning institutional practices. It is also important to transfer knowledge and purpose of a practice across boundaries in the institution. A further key element is to establish practices where multiple perspectives are heard and appreciated to ensure that the staff members can use opportunities to develop and experience themselves as acknowledged contributors to the institution. The current study, “Active Kindergarten – Active Children” (AK-AC), aims to examine the potential of a staff-led and expert-supported intervention to increase children’s PA level and reduce sedentary time within the ECEC setting compared to standard care.

The article "Children’s physical activity level and sedentary behaviour in Norwegian early childhood education and care: effects of a staff-led cluster-randomised controlled trial" was retracted in 2024. Reasons: results that could not be reproduced; errors in the methods; unreliable results or conclusions; concerns about the data.

## Methods

### Declarations

The AK-AC study was designed as a two-arm, randomised by ECEC institution, evaluative controlled trial with the overarching aim of increasing the children’s PA level and reduce sedentary time. The Regional Committee for Medical & Health Research Ethics found the research project to be outside the remit of the Act on Medical and Health Research; therefore, the study could be implemented without its approval (ref no. 2015/1034). Approval from the Norwegian centre for research data was given because no personal or sensitive information was collected or stored (ref no. 44760/3). Written consent was obtained from all parents based on both oral and written information about the project.

### Participants

All children attending one of the 11 public ECEC institutions in Sandefjord municipality and born in 2011 (3 or 4 year olds) (*n* = 130) were invited to participate in the study. Parents of a total of 116 children (89%) signed the informed consent form and children of these parents where included in the study. Figure 1 provides an overview of participant flow through the study. Intervention and control group was formed at the centre level; six ECEC institutions were randomly assigned to intervention group and five institutions to the control group. The ECEC institutions varied in size and number of children (range 28 children to 100 children). Most ECEC institutions follows the national recommended staff-child ratio of one staff member per three children under the age of three, and per six children over the age of three. Regulation also demand educated ECEC teacher per nine children under the age of three, and per 18 over the age of three. The distribution showed a mixture of centre size in both the intervention and control group.

The article "Children’s physical activity level and sedentary behaviour in Norwegian early childhood education and care: effects of a staff-led cluster-randomised controlled trial" was retracted in 2024. Reasons: results that could not be reproduced; errors in the methods; unreliable results or conclusions; concerns about the data.

**Fig. 1:** Flow of participants through the trial

### Intervention

Four PA experts (researchers (PhD) within the field of PA and health in children, and physical education teachers) in collaboration with two members of the ECEC staff and two members of the municipality health department (paediatric physiotherapists) developed a frame for the intervention based on COP elements to be further developed, concretized and implemented by the staff. The intervention lasted for 4 months and contained the following components (Table 1): pre-meetings and follow up meetings in each ECEC institution; start up seminar and two follow up courses with all the staff members; ongoing planning and collective reflections practice in the ECEC institutions; Facebook group; and an equipment-package.

**Table 1:** The components, dosage and a brief description of the content of the intervention based on the theory of Communities of Practice [35]

Intervention component	Dose	Description
Pre-meetings in each kindergarten	1 h	Information about project
Information brochure to parents		Information about project
Start-up seminar	6 h	• Lecture; Physical activity in the ECEC setting • Discussing baseline data and outdoor areas with each ECEC • Practical session with different play activities • Each ECEC institution developed an intervention program tailored to their institution, based on research and data from baseline. Focus on: staffs attitudes, knowledge, skills and competences and organization/environment
Two courses with 2 month intervals	3 + 3 h	Lecturing and discussion of self-determination theory. Practical sessions, sharing examples
Planning and implementation in each kindergarten	4 months	The ECEC institutions implemented their program
Detailed planning of daily physical activity activities	Weekly	Documentation of planned physical activity in weekly schedule
Reflections on how to promote physical activity	Regular	Reflection on who to promote physical activity were documented and discussed in each ECEC institution
Follow-up meetings in each kindergarten 1 month after start up seminar	1 h	• Supporting planning and implementing by project team • Practical session; example of physical activities and sharing of ideas • Discussions o How does the ECEC institution of your dreams look like? o What can you do to increase physical activity among the children?
Facebook group	4 months	Networking between ECEC institutions for ideas and inspiration
Equipment	1000 EUR	Equipment for physical active play and sweaters with logo for staff

### Measurements

The baseline measurements were conducted in September 2015 and the follow-up measurements immediately after the end of the intervention, May 2016. PA was assessed using ActiGraph GT3X+ accelerometers (ActiGraph, LLC, Pensacola, FL, USA). The children wore the accelerometer on the left hip during their stay at the ECEC setting for five consecutive days (Monday morning to Friday afternoon) on both time points. The staff attached the named monitors to the children every morning when they arrived at the ECEC institution and removed it at the end of each day. In order to ensure compliance with wearing the monitor, the staff were also instructed to make sure the monitor was fastened properly at all times and in the right position. The epoch length (sample interval) was set to 15 s [36] and reintegrated to 60s epochs, as recommended ([37]). In the analysis of accelerometer data, consecutive strings of epochs with a count value of zero lasting at least 60 min (with two exceptions) were treated as non-wear and thus removed from the data array [38]. Analyses were restricted to participants who wore the accelerometer for a minimum of 6 h per day on at least 2 days. Accelerometer data were downloaded using Actilife (version 6 from Actigraph) and further processed and analyzed using a specialized accelerometer analytical software (Kinesoft, version 3.3.80, Saskatchewan, Canada). The time (minutes) spent in various levels of PA intensity were calculated according to the cut-offs set by Butte et al. (2014), in which sedentary behaviour (sedentary time) was defined as ≤239 counts, light intensity PA was defined as 240 to 2119 counts, MVPA was defined as 2120 to 4449 counts, and any amount above 4450 was considered vigorous or very vigorous intensity PA [37]. We also calculated whether the children reached the PA recommendations of 60 min of MVPA per day [39].

The article "Children’s physical activity level and sedentary behaviour in Norwegian early childhood education and care: effects of a staff-led cluster-randomised controlled trial" was retracted in 2024. Reasons: results that could not be reproduced; errors in the methods; unreliable results or conclusions; concerns about the data.

### Statistical analysis

All statistical analyses were performed using SPSS (Statistical Package for the Social Sciences for Windows, version 24, IBM, Inc., Chicago, USA). Visual inspection of histograms and values of skewness and kurtosis indicated that all data were normally distributed. Descriptive data are presented as proportion, mean, and standard deviation (SD) with 95% confidence intervals (CIs) where appropriate. Within- and between-differences of interval data were evaluated by *t-*tests (independent *t-*tests and paired *t-*tests). Delta PA scores (T1-T0) were calculated and used as the dependent variable in the analysis of covariance (ANCOVA), with baseline measurements, age, wear time and sex as covariates when calculating the significance of differences between the groups. Odds ratios and 95% confidence intervals (CI) were computed from logistic regression using PA recommendations as the dependent variable, group as the primary independent variable and with age, gender and wear time as covariates. The 50% least physically active children and the 50% most physically active were defined by 50% lowest and highest total counts per min (CPM) on baseline, respectively. When analysing differences between the least and most active, adjustments were made for wear time, gender and age. The results are presented as mean differences between the two groups ± CI. All tests were based on two-sided probability.

The article "Children’s physical activity level and sedentary behaviour in Norwegian early childhood education and care: effects of a staff-led cluster-randomised controlled trial" was retracted in 2024. Reasons: results that could not be reproduced; errors in the methods; unreliable results or conclusions; concerns about the data.

## Results

The children were on average 3.7 years old (SD ± 0.4) at baseline, and 57 % were girls. There were no differences between the intervention and control groups on any of the PA variables at baseline. After excluding participants with unusable accelerometer data (*N* = 15), a final sample of 101 children was included in the analyses (77.7% of children assessed for eligibility) (see Fig. 1 for more details). Excluded participants were equally distributed between groups and did not differ in age, sex or PA level compared to included participants.

Except for vigorous intensity, the intervention group increased significantly more on all PA variables (Table 2). Adjusted for wear time and other potential confounders the intervention group increased their weekly time spent in MVPA by 50 min, took approx. 10,000 more steps and reduced sedentary time by 70 min compared to the control group.

**Table 2:** Physical activity level and sedentary time at baseline and follow-up for the two groups

	Intervention group		Control group				
	Baseline (*n* = 64)	Follow-up (*n* = 60)	Baseline (*n* = 47)	Follow-up (*n* = 41)	Adjusted ∆ diff (95 ± CI)^a^	Partial eta squared (η_p_^2^)	*P*-value^b^
Wear days	4.3 (0.8)	4.0 (1.1)	4.4 (0.8)	3.9 (1.2)	0.5 (−0.1, 1.0)		0.09
Wear time (min/day)	451 (36)	455 (42)	459 (39)	453 (48)	82 (− 8133)		0.06
Total PA level (CPM)	818 (243)	1118 (272)	807 (210)	989 (273)	118 (8228)	0.045	0.03
Light PA (Min/day)	160 (26)	171 (24)	168 (24)	167 (23)	13 (4,23)	0.07	< 0.01
MVPA (min/day)	58 (20)	74 (24)	58 (21)	66 (23)	10 (3,18)	0.07	0.01
Mod PA (min/day)	45 (15)	54 (16)	46 (17)	50 (16)	8 (2,13)	0.08	< 0.01
Vig PA (min/day)	13 (7)	20 (9)	12 (5)	16 (8)	2.7 (−1,6)	0.02	0.1
Steps per day	6652 (1421)	9063 (1681)	7365 (1601)	7956 (2148)	1909 (1130,2688)	0.2	< 0.01
Sed time (min/day)	265 (39)	210 (34)	264 (55)	218 (34)	−14 (−27,-1)	0.04	0.04

Values are mean SD, *PA* physical activity, *CPM* counts per minute, *Mod* moderate, *Vig* vigorous, *Sed* sedentary

^a^All variables were adjusted for their respective baseline value, age, wear time and gender

^b^ The adjusted delta differences between groups is significant at the 0.05 level

There was an increase in the number of children meeting the PA recommendations of ≥60 min of MVPA per day at follow-up compared to baseline for both the intervention group (47%) and the control group (25%) (Fig. 2). The intervention group had a 2.4 higher odds (95% CI = 1.05, 5.7; *P* = 0.04) of meeting the PA recommendations compared to the control group at follow-up.

The article "Children’s physical activity level and sedentary behaviour in Norwegian early childhood education and care: effects of a staff-led cluster-randomised controlled trial" was retracted in 2024. Reasons: results that could not be reproduced; errors in the methods; unreliable results or conclusions; concerns about the data.

**Fig. 2:** Percentage of children in the two groups meeting PA recommendations at baseline and follow-up

The intervention group increased their PA level from baseline to follow-up at all time points except early morning and during food breaks (11 and 14 o’clock) while the control group only significantly increased their PA level at 11 and 14 o’clock (Fig. 3). Compared to the control group, the increment from baseline to follow-up was significantly larger in the intervention group at hours 09–10 (mean diff. 331 CPM, 95% CI = 600, 62; *P* = 0.01), 10–11 (mean diff. 364, 95% CI = 202, 527; P < 0.01), 13–14 (mean diff. 241, 95% CI = 44, 438; *P* = 0.01) and 15–16 (mean diff. 362, 95% CI = 66, 658; *P* = 0.01).

**Fig. 3:** Delta (follow-up – baseline) physical activity level hour-by-hour for both groups

The 50% least active children on baseline in the intervention group increased MVPA by 14 min per day (95% CI = 5, 22, *P* < 0.01) more than the 50% least active children in the control group (Fig. 4). Furthermore, the 50% least active in the intervention group had a significantly greater increase in total PA level (mean diff. 23, 95% CI = 4, 44; *P* = 0.02) and steps per day (mean diff. 1936, 95% CI = 1124, 2749; P < 0.01) than the 50% least active children in the control group. Both groups reduced sedentary behavior, but there were no statistical difference between the two groups concerning sedentary time (Fig. 4). For the 50% most active children, those in the intervention group significantly reduced sedentary time (mean diff. -17 min, 95% CI = − 2, − 32; *P* = 0.02), but not MVPA, compared to the 50% most active in the control group (Fig. 4). Except for steps per day (mean diff. 1738, 95% CI = 449, 3026; *P* = 0.01) no other differences were found between the most active children in the two groups. The 50% least active children in the intervention group increased total PA level by 38% (95% CI = 19, 58; *P* < 0.01), MVPA by 12 min/day (95% CI = 2, 22; *P* = 0.02) and steps per day by 1228 (95% CI = 431, 2024; *P* < 0.01) more than the 50% most active in the intervention group. There were no differences in changes in sedentary time between the two subgroups. In the control group, there were no delta differences on any of the PA variable between the least and most active children.

**Fig. 4:** Delta differences (follow-up – baseline) for MVPA and sedentary time for the 50% least active and 50% most active at baseline in the intervention group (left) and control group (right)

The article "Children’s physical activity level and sedentary behaviour in Norwegian early childhood education and care: effects of a staff-led cluster-randomised controlled trial" was retracted in 2024. Reasons: results that could not be reproduced; errors in the methods; unreliable results or conclusions; concerns about the data.

## Discussion

The intervention increased three to four-year-old children’s total PA level, step count, time spent in light- and moderate intensity, and reduced sedentary time during their stay in the ECEC setting. By that, the number of children adhering to the PA recommendations increased significantly. Especially encouraging was that the least physically active at baseline gained the most from the intervention. The lack of effect on vigorous intensity PA can possibly be explained by the fact that the preschools, according to their self-developed plans, did not have specific goals of influencing this behaviour. The staff rather focused on routines, environment, games, plays and activities that targeted the general PA level, moderate intensity and sedentary time. Examples of interventions components are PA integrated in other everyday themes, establish more indoor space for activity, more use of the outdoor environment and more sensibility to see and support the least physically active children. It might also be explained by an underestimation of minutes spent in vigorous PA since we used 60s epochs and not 10s or 15 s epochs. Most children do not attain or sustain high levels of physical exertion for extended periods, and thus the use of 10–15 s epochs in the current study might have provided different results with regard to vigorous intensity PA. Although vigorous intensity PA is an interesting variable to look at, the collapsed category of MVPA may be more meaningful for health outcomes. Furthermore, the PA guidelines for children under five do not distinguish between moderate- and vigorous PA [39]. The baseline data were in line with findings from other studies indicating an insufficient degree of PA in children in ECEC settings [1, 2, 40]. The findings in this study are important because most children (83.5 and 97.1% of children between 1 and 2 and 3–5 years of age respectively) attend ECEC settings most days of the week, mostly for more than 40 h per week [16]. An effective intervention will thus benefit children across the socioeconomic spectrum.

An increase in the number of children adhering to the PA recommendations is important although we are only starting to understand the dose-response relationship of PA with health parameters in young children [41, 42]. However, there are some studies indicating increased PA can cause long time effects in terms of lower blood pressure [43] and improved aerobic fitness and cardiovascular health as well as decrease body fat [44, 45]. Hence, although we did not measure cardiovascular disease risk factors in this study, the results may be clinically important. The main objective in this study was to look at differences in PA level between the groups during their stay in the ECEC setting, including number of children achieving the PA recommendations, and not whether they adhered to the PA recommendations per se. To calculate the number of children reaching the PA recommendations one would have to measure PA throughout the week and not just during their stay in the ECEC setting. Our data is thus an underestimation of number of children adhering to the PA recommendations.

The article "Children’s physical activity level and sedentary behaviour in Norwegian early childhood education and care: effects of a staff-led cluster-randomised controlled trial" was retracted in 2024. Reasons: results that could not be reproduced; errors in the methods; unreliable results or conclusions; concerns about the data.

It is of particular interest, that these effects have been achieved through a staff-led intervention. As such, our results are contrasting studies that indicate no or only weak effects of staff-led interventions compared to the effects that has been achieved in some studies where the interventions was led by PA experts [20, 22, 24, 25, 46]. The explanation for these contrasting findings may be two folded. Firstly, a significant proportion (40%) of the about 93,000 staff in Norwegian ECEC services is trained as ECEC teachers, which means that they have higher education at least on a bachelor level and an additional 18% has relevant vocational education (child- and youth worker) [47]. Another 8% has higher education and 4% other forms of vocational education. This educational profile of staff indicates that staff, as least partly, has high competence in terms of both pedagogical and subject knowledge and, by this, is well suited to lead a PA intervention. This is in accordance with Finch et al. (2014) who have highlighted the importance of competence as a prerequisite for staff-led interventions [25]. Secondly, applying the collaborative and “bottom-up” Communities of Practice approach (COP; Wenger, 1999) might be particularly suited for Norwegian ECEC settings as both the national framework plan for ECEC teacher education [48] and the national framework plan for ECEC [49] emphasizes the importance of staff collaboration and organizational learning. Thus, a large proportion of the employees in ECEC settings might be sufficiently prepared to understand their organization as learning communities and capable of sharing competence and experiences to develop new practices. A high degree of professionalism and a combination of pedagogical and content knowledge relevant for facilitating PA in a collaborative and child cantered way might have been an important factor for understanding the findings in this study.

The fact that the intervention in the current study was collaborative and staff-led makes the results especially promising because, in comparison to expert-led programs, staff-led programs may be more cost-effective and easier to scale-up. Furthermore, this approach possibly increases the staff’s “sense of ownership” to the intervention and building a more autonomous organization, making it more likely that the institution will carry on focusing on PA once the research project ends, and succeed in this important work. As MacDonald and Green [34] highlighted, a dialogical and bottom up approach will take into account the specific context as well as differences within and between ECEC settings relevant for the promotion of physically active play and, by that, have the potential to be successful.

The article "Children’s physical activity level and sedentary behaviour in Norwegian early childhood education and care: effects of a staff-led cluster-randomised controlled trial" was retracted in 2024. Reasons: results that could not be reproduced; errors in the methods; unreliable results or conclusions; concerns about the data.

This study has some significant strengths and some important limitations. Strengths include a rigorous research design, objective measurement of PA and high attendance rate. The fact that almost all of the children that were eligible for the study agreed to wear an accelerometer on two occasions strengthens the generalizability of the study. This is an important point for this kind of studies, because the least physically active individuals, hence those we want to target the most, tend not to volunteer for studies of this nature. Further, a major strength of the study was that it was guided by PA experts but led by staff in each of the ECEC institutions. This flexible and pragmatic approach taken is most likely less costly than expert-driven programs, easier to scale-up and probably more likely to be continued after the research project ends. A limitation of this study is that we are not able to specifically evaluate the contribution of each of the intervention components and by that, assess which one were the most effective or feasible. Furthermore, a lack of process evaluation makes it difficult to determine to what degree the ECEC institutions followed the strategy laid out in the logic model. Furthermore, although we were successful in creating immediate post-program results, a lack of long-term follow-up leaves the question of whether the programme is effective in the long run.

## Conclusions

Our results show that a flexible staff-led and expert-supported multicomponent PA intervention can increase total PA level, MVPA and reduce time spent sedentary in three to four-year-old children during their stay in ECEC settings. Instead of purely implementing structured programs developed by external experts to increase physical active play in ECEC institutions, the findings from the current study indicate that there is a potential for interventions that emphasize collaborative reflection pedagogical practice between staff members for improvement of complex practice.

The article "Children’s physical activity level and sedentary behaviour in Norwegian early childhood education and care: effects of a staff-led cluster-randomised controlled trial" was retracted in 2024. Reasons: results that could not be reproduced; errors in the methods; unreliable results or conclusions; concerns about the data.

## Data Availability

Data can be accessed upon request. Contact person is Eivind Andersen, Eivind.andersen@usn.no

## Abbreviations

ECEC: early childhood education and care
PA: physical activity
MVPA: moderate- to vigorous intensity physical activity
COP: communities of practice
CI: confidence interval
AK-AC: Active Kindergarten – Active Children
SD: standard deviation
